# Application of Multimode Health Education Combined with Humanistic Care in Pain Management of Patients with Femoral Fracture and Its Influence on VAS Score

**DOI:** 10.1155/2021/1242481

**Published:** 2021-12-13

**Authors:** Ming Shi, Pengyu Zhang, Ling Xia, Zhiteng Wei, Fangjie Bi, Yujia Xu, Pan Wang

**Affiliations:** ^1^Department of Orthopedic, Zibo Central Hospital, Zibo 255000, Shandong Province, China; ^2^Department of Orthopedic, Zhangqiu District People's Hospital, Jinan 250200, Shandong Province, China; ^3^Department of Rehabilitation Medicine, Zibo Central Hospital, Zibo 255000, Shandong Province, China; ^4^Department of Orthopedic, Weifang Hospital of Traditional Chinese Medicine, Weifang 262699, Shandong Province, China; ^5^Department of Internal Medicine-Cardiovascular, Zibo Central Hospital, Zibo 255000, Shandong Province, China; ^6^Department of Ultrasonography, Zibo Central Hospital, Zibo 255000, Shandong Province, China; ^7^Department of Pain, Zibo Central Hospital, Zibo 255000, Shandong Province, China

## Abstract

**Objective:**

To explore the application of multimode health education combined with humanistic care in pain management of patients with femoral fracture and its influence on VAS score.

**Methods:**

A total of 120 patients with femoral fracture admitted in our hospital (May 2017–May 2021) were selected as the research objects. The patients who received routine health education were included into the routine group, and the patients who received multimode health education combined with humanistic care were included into the combined group, with 60 cases in each group. The pain management effect of the two groups was compared after nursing intervention.

**Results:**

No significant difference was found in age, BMI, fracture sites, gender, education degree, and residence between the two groups (*P* > 0.05). The awareness rate of health knowledge of the combined group was as high as 93.33%, which was obviously higher than that of the routine group (*P* < 0.05). Compared with the routine group, excellent rates of sitting durability and joint range of motion in the combined group were obviously higher (*P* < 0.05), and poor rates of sitting durability and joint range of motion in the combined group were obviously lower (*P* < 0.05). Compared with the routine group, VAS scores of the combined group at 1 d, 2 d, and 3 d after admission and at 1 d, 2 d, and 3 d after surgery were remarkably lower (*P* < 0.05). Compared with the routine group, compliance of exercise, medical waist belt using, and working posture of the combined group 1 week, 1 month, and 6 months after surgery was obviously higher (*P* < 0.05). Compared with the routine group, the scores of Rasmussen and Johner-Wruhs of the combined group 6 months after surgery were conspicuously higher (*P* < 0.05).

**Conclusion:**

The application of multimode health education combined with humanistic care in pain management of patients with femoral fracture can effectively relieve pain, improve the awareness rate of health knowledge, promote the recovery of lower limb function, and enhance the prognosis of quality of life for patients.

## 1. Introduction

Pain is a common and unavoidable clinical feature in orthopedic perioperative period, and severe pain results in a series of serious complications, which affect the treatment effect and prognosis of functional recovery in the perioperative period. Therefore, more and more attention is paid to pain management of orthopedic patients in clinics. Meanwhile, pain has become the fifth vital sign after body temperature, pulse, respiration, and blood pressure. Therefore, pain management of orthopedic patients is of great significance in improving the treatment effect and prognosis of quality of life [1–3]. According to clinical experience of the author, femur fractures are mostly caused by external trauma. The treatment effect of the disease and the medical compliance are directly affected by perioperative psychological status of patients, awareness of the disease, trust in physicians, and pain management effects. The subject of clinical nursing service is human, who is the unique individual with complex emotions. In this way, the nursing service should not only treat with scientific and professional symptomatic measures but also provide respect, understanding, and care. Clinical statistics found that with the development of orthopedic health education activities, single oral and written education is having difficulty in satisfying the needs of patients and their family members, and less conducive to mobilizing the initiative and enthusiasm of their participation in medical activities, whereas multimode health education, which breaks the traditional education, is able to combine factors such as oral explanation, video guidance, and model reference to promote the novelty and diversity of health education. In addition, the integration of the novel concept of humanistic caring can shift the focus of nursing from disease to patient, which is good for improving the level of clinical nursing. Therefore, it is believed that multimode health education combined with humanistic care plays an essential role in the nursing of patients with femoral fracture, but at present, the combination of the two in orthopedic traumatic diseases has rarely been studied. The research results are as follows.

## 2. Materials and Methods

### 2.1. Screening and Grouping

A total of 120 patients with femoral fracture admitted in our hospital (May 2017–May 2021) were selected as the research objects. The patients who received routine health education were included into the routine group, and the patients who received multimode health education combined with humanistic nursing were included into the combined group, with 60 cases in each group. The study was approved and supervised by the hospital ethics committee.

### 2.2. Inclusion Criteria

The exclusion criteria were as follows. Patients met the diagnosis of femoral fracture [4] and were confirmed by imaging examination. Patients had clear awareness and could be communicated with. Patients had no cognitive impairment. Patients and their family members understood the purpose, process, and significance of the study and signed the consent form.

### 2.3. Exclusion Criteria

The exclusion criteria were as follows. Patients had severe and unstable conditions. Patients presented with coma and shock. Patients were complicated with other organic diseases, systematic diseases, and malignant tumors. Patients were complicated with fracture of other sites. Patients had pathological fracture. Patients had poor medical compliance. Patients did not have complete medical records. Patients were complicated with other unstable underlying diseases.

### 2.4. Methods

In the routine group, patients were given routine health education at three important time points, i.e., at the time of admission, during perioperative period, and after discharge, mainly in the form of one-to-one oral education or education in writing; meanwhile, routine nursing measures were performed based on the clinical manifestations of patients with femoral fracture according to the medical advice [5, 6].

Based on the routine group, various education modes were applied for the combined group, including written education, media education, demonstration education, and collective education, together with humanistic care, so as to improve the participation of patients and to establish an effective health education program for pain management. The health education group was established, with clarified responsibility, to formulate the health education program for pain management, which centered on patients and their family members [7–9]. The targeted training should be organized for the application of humanistic care in medicine, the body influence of pain, the pain performance, analgesic methods, analgesic efficacy, and pain cognition. Through the analysis of clinical cases, the professional skills of nursing staff should be improved, and the role of humanistic care should be further clarified. The patients were evaluated comprehensively after admission. The nursing staff were required to kindly discuss over sleep and pain perception with the patients, carry out health education with common words, mainly consisting of the causes of perioperative pain, the influence of pain on body, and the significance and methods of analgesia, and answer the questions of patients in time. Moreover, nurses should map out appropriate plans for perioperative pain management combined with the advice of family members of patients and actively give feedback to medical staff about degree of pain control and other conditions. The one-to-one individualized mode was the most direct and common way in the health education. Nurses could give individualized guidance according to the specific conditions of patients, so as to better understand the psychological state of patients and solve patients' personal problems face to face. Written education resorted to health education manuals or cards with words and pictures, which mainly included femoral fracture rehabilitation knowledge, complications prevention and treatment, diet and exercise guidance. It was also a traditional education mode more convenient for consultation anytime to deepen patients' health knowledge. Media education was to present the key health knowledge to the patients and their families visually and vividly through the closed-circuit television and multimedia, presenting high degree of acceptance and leaving deep impression on patients and their family members. In the process of treatment and recovery, patients with femoral fracture were in need of limb exercise and the use of some instruments and crutches. Demonstration education required nursing staff to improve the patients' mastery of health knowledge and skills through personal demonstration and hand-to-hand teaching, which could effectively improve the patients' self-care ability [10–12]. Collective education was more comprehensive and more flexible, which could not only improve the efficiency of education but also facilitate the communication between patients and thus deliver a better effect combined with individualized education.

### 2.5. Observation Indexes

The general data including age, BMI, fracture sites, gender, education degree, and residence were recorded at admission. Awareness rate of health knowledge was evaluated by the questionnaire of health knowledge formulated by our hospital, which was distributed to the patients with femoral fracture 3 days before discharge, with a total score of 100 points. The scale had better stability, structure validity, and criterion validity. Patients and their family members should be informed of the purpose and significance of the survey, and the patients should fill in the questionnaire by themselves to ensure the authenticity and accuracy. The scores of more than 60 points indicated qualified.

Sitting durability of patients was evaluated before discharge, which was divided into four grades as poor, average, good, and excellent. Meanwhile, range of motion of joints was evaluated before discharge, which was divided into the same four grades. The incidence was calculated and compared in line with the corresponding grade between both groups.

The pain degree of patients at 1 d, 2 d, and 3 d after admission and at 1 d, 2 d, and 3 d after surgery was evaluated according to the visual analogue scale (VAS) score. A vernier marked with 0–10 points was used for assessment. 0 points indicated painless, and 10 points indicated the most severe pain that was unbearable. Higher scores indicated higher degree of pain. The compliance behavior of patients with femoral fracture was evaluated by using a self-made compliance questionnaire at 1 week, 1 month, and 6 months after surgery, which included exercise, medical waist belt using, and correct working posture.

At 6 months after surgery, recovery of lower limb function of patients with femoral fracture was reexamined by Rasmussen score for knee function [13] (0–30 points) and by Johner-Wruhs score for ankle function [14] (0–100 points). The higher the score, the better the knee or ankle function of patients.

### 2.6. Statistical Processing

All statistical data of the study were processed by SPSS 22.0 to calculate the difference between groups, and the pictures were graphed by GraphPad Prism 7 (GraphPad Software, San Diego, USA). Including enumeration data and measurement data in the form of (*n* (%)) and (‾*x* ± *s*), respectively, the study used the *X*^2^ test and *t*-test. The differences were statistically significant at *P* < 0.05.

## 3. Results

### 3.1. General Data

After comparison of the general data of both groups, no significant difference was found in age, BMI, fracture sites, gender, education degree, and residence (*P* > 0.05) (Table 1).

### 3.2. Awareness Rate of Health Knowledge

The awareness rate of health knowledge of the combined group was as high as 93.33%, which was obviously higher than that of the routine group (*P* < 0.05), with statistical significance (Figure 1).

### 3.3. Sitting Durability and Joint Range of Motion

Compared with the routine group, excellent rates of sitting durability and joint range of motion in the combined group were obviously higher (*P* < 0.05), and poor rates of sitting durability and joint range of motion in the combined group were obviously lower (*P* < 0.05) (Tables 2 and 3).

### 3.4. VAS Scores

Compared with the routine group, VAS scores of the combined group at 1 d, 2 d, and 3 d after admission and at 1 d, 2 d, and 3 d after surgery were remarkably lower (*P* < 0.05) (Figure 2).

### 3.5. Comparison of Compliance

Compared with the routine group, compliance of exercise, medical waist belt using, and correct working posture of the combined group 1 week, 1 month, and 6 months after surgery was obviously higher (*P* < 0.05) (Table 4).

### 3.6. Lower Limb Function

Compared with the routine group, the scores of Rasmussen and Johner-Wruhs of the combined group 6 months after surgery were conspicuously higher (*P* < 0.05) (Figure 3).

## 4. Discussion

### 4.1. Effect of Multimode Health Education Combined with Humanistic Care on Pain Management of Patients with Femoral Fracture

Femoral fracture is mostly caused by trauma, which is similar to the clinical manifestations of common fracture. However, femoral fracture is mainly characterized by trauma, severe pain, shock, and even other more serious systemic diseases [15, 16]. Patients with femoral fracture usually suffer from severe pain and fear, which may aggravate body stress response, increase the risk of complications, and thus affect recovery. Therefore, accurate assessment is the first step in pain management, which can provide effective information for pain control, and also help to evaluate the effect of pain treatment [17–19]. Multimode health education combined with humanistic care can help patients to eliminate fear from multiple dimensions, improve their psychological threshold of pain, and be aware of pain control measures, so that they can better cooperate with the treatment. Before health education for the combined group, the nurses discussed with each patient to identify their individual needs of pain management and implemented targeted education and guidance for patients. The results showed that the awareness rate of health knowledge of the combined group was as high as 93.33%, which was obviously higher than that of the routine group (*P* < 0.05), which was in line with the study of Anita J. Meehan et al. [20]. Compared with the routine group, VAS scores of the combined group at 1 d, 2 d, and 3 d after admission and at 1 d, 2 d, and 3 d after surgery were remarkably lower (*P* < 0.05). It indicated that multimode health education combined with humanistic nursing could better disseminate health knowledge and improve patients' awareness of femoral fracture to overcome their fear and build confidence, which made pain management more humanized, scientific, and comprehensive and served as the safeguard for implementation of pain management.

### 4.2. Effect of Multimode Health Education Combined with Humanistic Care on Compliance of Patients with Femoral Fracture

The results showed that compared with the routine group, compliance of exercise, medical waist belt using, and working posture of the combined group 1 week, 1 month, and 6 months after surgery was obviously higher (*P* < 0.05). This result confirmed that health knowledge education could work on in short term, especially when patients were seriously ill or had severe pain, so the compliance was high. However, with the extension of postoperative time and less discomfort symptoms, patients in the routine group tended to ignore the limb function exercise and daily life precautions. While, patients in the combined group had better adherence in a longer period, indicating that this intervention method was more comprehensive and effective, which also reflected the significance in the postoperative nursing. Postoperative compliance behaviors of effective functional exercise, wearing waist belt, and correct working posture lay the foundation for femoral healing, which can reduce waist and leg pain, strengthen the stability of spinal stabilization, and prevent recurrence. According to the study of Yeh Hsiang Fen et al. [21], the recurrence rate of waist and leg pain in patients with femoral fractures is 10.06%, which is attributed to lack of correct exercise of limb function during the critical period of postoperative recovery. Thus, postoperative limb function exercise is all the more necessary for patients with femoral fracture. After comparison of the clinical data of the two groups, it is clear that the compliance of patients is changeable, and the longer the time, the lower the compliance. Reduced compliance of the routine group is more obvious, so after carrying out effective health education, how to establish a long-term effective follow-up mechanism and system is a key issue in clinical practice, and their effect on patients should be continuously explored in subsequent related studies.

### 4.3. Effect of Multimode Health Education Combined with Humanistic Care on Functional Recovery of Patients with Femoral Fracture

Health education is one of the most effective and the primary steps to promote rehabilitation for patients with femoral fracture and is also an important method to improve health of patients [22, 23]. The multimode health education combined with humanistic care helps to change the health concept and health behavior of patients, coordinate the nurse-patient relationship, promote the early recovery, reduce complications, and reduce the disability rate. As femur is the largest bone in the whole body, fracture leads to serious condition with slow recovery and long hospitalization time, which is difficult for nursing and easily triggers multisystem complications. Therefore, in the clinical health education of femoral fracture, the concept of humanistic care should be put into application, with the dissemination of orthopedic knowledge as the breakthrough point, through multimode intervention, so as to achieve education that is early implemented, all-round, targeted, planned, random, continuous, and point-to-area [24, 25]. At the same time, the health education for family members is also important because with the support of them, the essence of patient-centered overall nursing can be truly reflected, so that patients can benefit for a long time. In addition, a health education mode including guidance, joint discussion, cooperation, and participation should be established, which should pay more attention to patients' feedback, and the nursing intervention plan can be adjusted timely, so as to ensure the rapid recovery. The results showed that compared with the routine group, excellent rates of sitting durability and joint range of motion in the combined group were obviously higher (*P* < 0.05), and poor rates of sitting durability and joint range of motion in the combined group were obviously lower (*P* < 0.05). Compared with the routine group, the scores of Rasmussen and Johner-Wruhs of the combined group 6 months after surgery were conspicuously higher (*P* < 0.05). It indicated that multimode health education combined with humanistic care delivered a positive effect on recovery of limb function for patients with femoral fracture, which was the safeguard for body rehabilitation.

To sum up, the application of multimode health education combined with humanistic care in pain management of patients with femoral fracture can effectively relieve pain, improve the awareness rate of health knowledge, promote the recovery of lower limb function, and enhance the prognosis of quality of life for patients.

## Figures and Tables

**Figure 1:** Comparison of awareness rate of health knowledge (%). The abscissa indicates groups, and the ordinate indicates the percentage (%). In the routine group, 44 cases were qualified, with the awareness rate of health knowledge of 73.33%. In the combined group, 56 cases were qualified, with the awareness rate of health knowledge of 93.33%. ^*∗*^Conspicuous difference in the awareness rate of health knowledge between the two groups (*X*^2^ = 8.640, *P* = 0.003).

**Figure 2:** Comparison of VAS scores between the two groups (‾*x* ± *s*). The abscissa indicates time nodes, and the ordinate indicates the score. The VAS scores of the routine group at 1 d, 2 d, and 3 d after admission and at 1 d, 2 d, and 3 d after surgery were (5.73 ± 0.86), (5.02 ± 0.61), (4.11 ± 0.65), (5.58 ± 0.73), (4.38 ± 0.66), and (3.52 ± 0.55). The VAS scores of the combined group at 1 d, 2 d, and 3 d after admission and at 1 d, 2 d, and 3 d after surgery were (4.81 ± 0.82), (4.15 ± 0.58), (3.27 ± 0.60), (4.77 ± 0.66), (3.85 ± 0.37), and (3.16 ± 0.42). ^*∗*^Significant differences in the VAS scores between the two groups at 1 d, 2 d, and 3 d after admission from left to right (*t* = 5.997, *t* = 8.001, *t* = 7.356, *P* < 0.001). ^#^Significant differences in the VAS scores between the two groups at 1 d, 2 d, and 3 d after surgery from left to right (*t* = 6.375, *t* = 5.426, *t* = 4.030, *P* < 0.001).

**Figure 3:** Comparison of the scores of Rasmussen and Johner-Wruhs. The abscissa indicates evaluation dimensions, and the ordinate indicates the scores. The scores of Rasmussen and Johner-Wruhs in the routine group were (24.55 ± 3.16) and (84.79 ± 3.18). The scores of Rasmussen and Johner-Wruhs in the combined group were (28.24 ± 1.57) and (95.57 ± 1.41). ^*∗*^Significant difference in Rasmussen scores between the two groups (*t* = 8.100, *P* < 0.001). ^*∗∗*^Significant difference in Johner-Wruhs scores between the two groups (*t* = 24.005, *P* < 0.001).

**Table 1:** Comparison of general data (*n* = 60).

Observation indexes	Routine group	Combined group	X^2^/*t*	*P*
Age (years old)	54.68 ± 5.36	55.21 ± 5.42	0.539	0.591
BMI (kg/m^2^)	23.46 ± 3.17	23.51 ± 3.22	0.086	0.932

Fracture sites				
Fracture of proximal femur	23 (38.33)	22 (36.67)	0.036	0.850
Femoral shaft fracture	16 (26.67)	18 (30)	0.164	0.685
Distal femoral fracture	21 (35)	20 (33.33)	0.037	0.847

Gender			0.333	0.564
Male	41 (68.33)	38 (63.33)		
Female	19 (31.67)	22 (36.67)		

Education degree			0.137	0.711
High school degree below	36 (60)	34 (56.67)		
Junior high school degree and above	24 (40)	26 (43.33)		

Residence			0.134	0.714
Urban	31 (51.67)	33 (55)		
Rural	29 (48.33)	27 (45)		

**Table 2:** Comparison of sitting durability between the two groups (*n* (%)).

Group	Poor	Average	Good	Excellent
Routine group (*n* = 60)	8 (13.33)	9 (15)	10 (16.67)	33 (55)
Combined group (*n* = 60)	1 (1.67)	5 (8.33)	6 (10)	48 (80)
*X* ^2^	5.886	1.294	1.154	8.547
*P*	0.015	0.255	0.283	0.003

**Table 3:** Comparison of joint range of motion between two groups (*n* (%)).

Group	Poor	Average	Good	Excellent
Routine group (*n* = 60)	9 (15)	19 (31.67)	18 (30)	14 (23.33)
Combined group (*n* = 60)	2 (3.33)	13 (21.67)	20 (33.33)	25 (41.67)
*X* ^2^	4.904	1.564	0.154	4.596
*P*	0.027	0.215	0.695	0.032

**Table 4:** Comparison of compliance behaviors (*n* (%)).

Evaluation indexes		Routine group	Combined group	*X* ^2^/*P*
Exercise	1 week	52 (86.67)	60 (100)	8.571/0.003
	1 month	47 (78.33)	55 (91.67)	4.183/0.041
	6 months	24 (40)	36 (60)	4.800/0.028

Medical waist belt using	1 week	50 (83.33)	58 (96.67)	5.926/0.015
	1 month	47 (78.33)	56 (93.33)	5.551/0.018
	6 months	32 (53.33)	43 (71.67)	4.302/0.038

Correct working posture	1 week	49 (81.67)	59 (98.33)	9.259/0.002
	1 month	46 (76.67)	57 (95)	8.292/0.004
	6 months	30 (50)	41 (68.33)	4.174/0.041

## Data Availability

The data used to support the findings of this study are available from the second author upon request.
